RETRACTED

# Prognostic and clinicopathological significance of C-reactive protein/albumin ratio (CAR) in patients with gastric cancer: A meta-analysis

**DOI:** 10.1371/journal.pone.0250295

**Published:** 2021-04-26

**Authors:** Junhua Yu, Huiling Liu, Xueyun Zeng, Yujun Zhao, Dejun Jiang, Hang Lu, Jun Qian

**Affiliations:** 1 Department of General Surgery, The Quzhou Affiliated Hospital of Wenzhou Medical University, People’s Hospital of Quzhou, Quzhou, Zhejiang, China; 2 Department of Pharmacy, Zhejiang Quhua Hospital, Quzhou, Zhejiang, China; Universitá Sapienza di Roma, ITALY

## Abstract

**Background:**

In recent years, many studies have explored the potential prognostic utility of C-reactive protein/albumin ratio (CAR) in patients with gastric cancer (GC), however, the results remain conflicting. We thus performed a meta-analysis to determine the association of CAR and prognosis of GC.

**Methods:**

This meta-analysis was conducted according to the Preferred Reporting Items for Systematic Reviews and Meta-Analyses (PRISMA) Statement. PubMed, Web of science, Embase, and Cochrane Library were searched. Hazard ratios (HRs) and 95% confidence intervals (CIs) for overall survival (OS) and cancer-specific survival (CSS) of included studies were pooled to estimate the prognostic value of CAR.

**Results:**

Eight studies with a total of 3,216 patients were included in this meta-analysis. High CAR was significantly associated with poor OS (HR = 1.59, 95%CI = 1.36–1.85, p<0.001) and worse CSS (HR = 1.65, 95%CI = 1.21–2.25, p = 0.002). In addition, high CAR was significantly associated with male sex (OR = 1.80, 95%CI = 1.31–2.47, p<0.001), advanced tumor stage (OR = 2.14, 95%CI = 1.48–3.09, p<0.001), and tumor size ≥3cm (OR = 2.69, 95%CI = 1.84–3.93, p<0.001).

**Conclusion:**

Elevated pretreatment CAR is a prognostic marker of poor OS and CSS in patients with GC. Furthermore, high CAR levels are associated with clinicopathological features reflecting tumor progression.

## Introduction

Gastric cancer (GC) is the fourth most commonly diagnosed cancer and the second leading cause of cancer-related death around the world [1]. GC is a global health burden and it is estimated that 1,033,701 new GC cases and 782,685 deaths occurred in 2018 worldwide [2]. The risk factors of GC include *H*. *pylori* infection, geographical location, socioeconomic status, and age [3]. Surgery is the only chance for curative treatment; and implementation of a multidisciplinary approach is mandatory and improves survival outcomes [4]. The prognosis of GC depends largely on the stage at initial diagnosis. The 5-year overall survival (OS) rate for patients with GC is 65% without metastases [3], whereas advanced disease carries a dismal prognosis with the median survival of 4–12 months and a 5-year OS rate <5% [4, 5]. Recent progress of treatment of GC improved the survival outcomes of patients. Immune checkpoint inhibitors (ICI) including nivolumab and pembrolizumab has been emerging as a novel treatment strategy for advanced GC [6]. Recent research points to CAR-T immunotherapy as a promising treatment for GC [7]. Prognostic markers including platelet count, CA 19–9, CEA, and neutrophil-to-lymphocyte ratio (NLR) are reported to be highly associated with prognosis of GC [8]. Because of poor prognosis of patients with late-stage, it is important to identify simple and useful biomarkers to help prognostic assessment and therapeutic modalities selection.

RETRACTED

Growing evidence has proven that inflammatory responses and nutritional status exert pivotal roles in carcinogenesis, progression, and metastasis of cancer [9–11]. C-reactive protein (CRP) is an acute phase marker of inflammation and is reported to associate with inferior prognosis in various cancers [12]. CRP is produced by hepatocytes, mainly in response to interleukin 6 (IL-6) secreted by T cells and macrophages, which regulates the production of CRP at the transcriptional level [13]. CRP is a sensitive marker of systemic inflammation [14]. Moreover, patients with cancer experience physical and metabolic effects of the disease, and inadequate food intake caused by anticancer treatment, often leads to the malnutrition state of patients [15]. Serum albumin (ALB) is an indicator of nutritional status and hypoalbuminemia suggests that the overall condition of patients is poor [16]. Recent studies report that the C-reactive protein/albumin ratio (CAR), as a novel inflammation biomarker, has shown independent prognostic effect in various types of cancer, including hepatocellular carcinoma [17], renal cell carcinoma [18], esophageal cancer [19], and colorectal cancer [20]. A recent study showed that CAR was an independent predictor for postoperative complications following gastrectomy of GC [21]. Another study indicated that CAR was strongly associated with poor prognosis in patients who underwent surgery for esophagogastric junction and upper gastric cancer (UGC). Many studies also investigated the association of CAR and prognosis in GC, with the results remain controversial [22–29]. Therefore, we aggregated data of eligible studies and performed a meta-analysis to quantify the prognostic role of CAR in GC.

## Materials and methods

### Literature strategy

This meta-analysis was conducted according to the Preferred Reporting Items for Systematic Reviews and Meta-Analyses (PRISMA) Statement [30]. The electronic databases of PubMed, Web of science, Embase, and Cochrane Library were comprehensively searched through 10 November 2019. The combinations of following text words and Medical Subjects Heading [MeSH] terms were used for search: (“C-reactive protein to albumin ratio” OR “C-reactive protein/albumin ratio” OR “CRP/Alb ratio” OR “C-reactive protein Albumin ratio”) AND (“gastric cancer” OR “gastric carcinoma” OR “stomach cancer” OR “stomach neoplasm”). The references list of included articles and recent reviews were also manually searched for potential eligible studies. Ethical approval was not required for this meta-analysis since all used data were extracted from previous publications and no personal data were involved.

RETRACTED

### Eligible criteria

The eligible studies must meet the following inclusion criteria: (1) GC was pathologically diagnosed; (2) pretreatment CAR was evaluated by serum-based methods; (3) the association between CAR and prognosis of patients including OS and/or cancer-specific survival (CSS) was estimated or sufficient data to calculate hazard ratios (HRs) and 95% confidence intervals (CIs) were provided; (4) a cut-off value of CAR was identified; (5) full-text published in English language. Exclusion criteria were as follows: (1) conference abstracts, reviews, letters, or case reports; (2) studies with insufficient data for analysis; (3) non-human studies; (4) duplicate studies.

### Data extraction and quality assessment

All studies were reviewed by two investigators (J.Y. and H.L.) independently, and all discrepancies were resolved by discussion. The extracted information included the following items: first author, year of publication, country, sample size, enrollment time, patient age, sex, tumor node metastasis (TNM) stage, study type, follow-up time, cut-off value, treatment, survival outcomes and HRs and 95%CIs. When univariate and multivariate analyses were both conducted, the data of multivariate analysis were extracted from included studies. The quality of included studies was evaluated according to Newcastle-Ottawa Scale (NOS) [31]. The NOS evaluates the quality of 3 perspectives: selection, comparability, and clinical outcomes, with a score ranging from 0 to 9. A study with a NOS score ≥6 is regarded as of high quality.

### Statistical analysis

The Stata SE 12.0 (Stata Corporation, College Station, TX, USA) was used to perform all calculations in this meta-analysis. HRs and 95%CIs for OS and CSS of included studies were pooled to estimate the prognostic value of CAR. The heterogeneity of all studies was assessed by using Cochran’s Q test and Higgins *I*^2^ test. When significant heterogeneity was observed (*I*^2^>50% and/or P<0.10), a random-effects model was used; otherwise, a fixed-effects model was adopted. The correlation of CAR and clinicopathological features was evaluated by pooling odds ratios (ORs) and 95%CIs. Subgroup analyses stratified by country, treatment, cut-off value, and TNM stage were performed. These confounders were extracted from each individual study included in this meta-analysis. Publication bias was evaluated using Begg’s test. A p<0.05 was identified as statistically significant.

RETRACTED

## Results

### Study selection process

The flowchart of study selection process is presented in Fig 1. Initial literature search identified 123 records; and after duplicates were removed, 92 records were screened. Based on titles and abstracts evaluation, 73 studies were excluded and 19 studies were further evaluated by full-text examination. Eleven full-text articles were excluded by the following reasons: 9 studies lacked sufficient data, 1 study was a duplicate study, and 1 study did not focus on GC. Finally, 8 studies with a total of 3,216 patients [22–29] were included in this meta-analysis.

**Fig 1:** Flow diagram showing study retrieval and selection process.

### Characteristics of included studies

The baseline characteristics of these 8 included studies were summarized in Table 1. All studies were conducted in Asia in two countries; 5 in China [22, 23, 25, 28, 29] and 3 in Japan [24, 26, 27]. The sample sizes ranged from 240 to 688; and the median value was 392.5. Six studies with 2,127 patients [22–27] reported the association between CAR and OS and 3 studies with 1473 patients [24, 28, 29] provided the data of CAR on CSS. Seven studies were of retrospective study design [22–28] and 1 study was a prospective study [29]. The cut-off values of CAR ranged from 0.0232 to 0.5897 in included studies. The NOS scores of included studies ranged from 6 to 9, with a median value of 7.5, indicating that all included studies were of high-quality.

**Table 1:** Characteristics of the studies included in this meta-analysis.

Author	Year	Country	Sample size	Age (years)	Sex (M/F)	Treatment	TNM stage	Types of outcomes	Cut-off value	Analysis	NOS score	Follow-up (months)	Study type	Study period
Liu	2015	China	455	59(19–86)	314/141	Surgery	I-III	OS	0.25	MV	7	25(1–76)	Retrospective	2005–2010
Ni	2016	China	258	NR	184/74	Chemotherapy	IV	OS	0.5897	MV	6	7(0.2–68)	Retrospective	2010–2015
Toiyama	2016	Japan	384	67(32–88)	264/120	Surgery	I-III	OS, CSS	0.051	MV	8	47.6	Retrospective	2001–2011
Mao	2017	China	337	59(19–89)	237/100	Mixed	I-IV	OS	0.3778	MV	6	NR	Retrospective	Jan-Dec, 2010
Saito	2018	Japan	453	NR	331/122	Surgery	I-IV	OS	0.0232	UV	6	61.9	Retrospective	2005–2013
Toyokawa	2018	Japan	240	64.5	168/72	Surgery	II	OS	0.03	MV	9	100.5	Retrospective	1997–2012
Liu	2019	China	688	57(21–86)	449/239	Mixed	II-III	CSS	0.2	MV	8	36(3–162)	Retrospective	2000–2012
Lu	2019	China	401	58.6	271/130	Surgery	I-III	CSS	0.143	MV	9	24(3–35)	Prospective	2015–2016

M, male; F, female; NR, not reported; OS, overall survival; CSS, cancer-specific survival; MV, multivariate; UV, univariate; NOS, Newcastle-Ottawa Scale; TNM, tumor node metastasis.

RETRACTED

### Correlation between pretreatment CAR and OS

A total of 6 studies involving 2,127 patients [22–27] explored the relationship of CAR and OS in GC. As shown in Fig 2 and Table 2, the combined results indicated that high CAR was significantly associated with poor OS (HR = 1.59, 95%CI = 1.36–1.85, p<0.001), with no significant heterogeneity (*I*^2^ = 0, P = 0.628). The subgroup analysis was carried out based on 3 variables: country, treatment, cut-off value, and TNM stage. As summarized in Table 2, the pooled data demonstrated that elevated CAR remained a significant marker of inferior OS irrespective of country, treatment, cut-off value, or TNM stage.

**Fig 2:** Forest plot of CAR in predicting OS of patients with GC. (A) The whole patients group; (B) The subgroup analysis by country; (C) The subgroup analysis by treatment; (D) The subgroup analysis by cut-off value; and (E) The subgroup analysis by TNM stage.

**Table 2:** The subgroup analyses for the association between CAR and OS and CSS in gastric cancer.

Subgroups	No. of studies	No. of patients	Fixed-effects model		Random-effects model		Heterogeneity	
			HR (95%CI)	p	HR (95%CI)	p	*I*^2^(%)	Ph
**OS**								
Total	6	2,127	1.59(1.36–1.85)	<0.001	1.59(1.36–1.85)	<0.001	0	0.628
Country								
China	3	1,050	1.51(1.26–1.80)	<0.001	1.51(1.26–1.80)	<0.001	0	0.414
Japan	3	1,077	1.86(1.36–2.55)	<0.001	1.86(1.36–2.55)	<0.001	0	0.811
Treatment								
Surgery	4	1,532	1.74(1.39–2.17)	<0.001	1.74(1.39–2.17)	<0.001	0	0.856
Mixed	1	337	1.78(1.20–2.65)	0.004	1.78(1.20–2.65)	0.004	-	-
Chemotherapy	1	258	1.33(1.03–1.73)	0.030	1.33(1.03–1.73)	0.030	-	-
Cut-off value								
<0.2	3	1,077	1.86(1.36–2.55)	<0.001	1.86(1.36–2.55)	<0.001	0	0.811
≥0.2	3	1,050	1.51(1.26–1.80)	<0.001	1.51(1.26–1.80)	<0.001	0	0.414
TNM stage								
I-III	2	839	1.73(1.31–2.28)	<0.001	1.73(1.31–2.28)	<0.001	0	0.386
IV	1	258	1.33(1.03–1.73)	0.030	1.33(1.03–1.73)	0.030	-	-
I-IV	2	790	1.79(1.30–2.45)	<0.001	1.79(1.30–2.45)	<0.001	0	0.977
II	1	240	1.71(1.02–2.87)	0.043	1.71(1.02–2.87)	0.043	-	-
**CSS**								
Total	3	1,473	1.65(1.21–2.25)	0.002	1.65(1.21–2.25)	0.002	0	0.919
Country								
China	2	1,089	1.58(1.09–2.29)	0.015	1.58(1.09–2.29)	0.015	0	0.923
Japan	1	384	1.82(1.03–3.22)	0.040	1.82(1.03–3.22)	0.040	-	-
Treatment								
Surgery	2	785	1.76(1.05–2.95)	0.033	1.76(1.05–2.95)	0.033	0	0.775
Mixed	1	688	1.59(1.08–2.35)	0.019	1.59(1.08–2.35)	0.019	-	-
Cut-off value								
<0.2	2	785	1.76(1.05–2.95)	0.033	1.76(1.05–2.95)	0.033	0	0.775
≥0.2	1	688	1.59(1.08–2.35)	0.019	1.59(1.08–2.35)	0.019	-	-
TNM stage								
I-III	2	785	1.76(1.05–2.95)	0.033	1.76(1.05–2.95)	0.033	0	0.775
II-III	1	688	1.59(1.08–2.35)	0.019	1.59(1.08–2.35)	0.019	-	-

RETRACTED

### Association of pretreatment CAR and CSS

Three studies enrolling 1473 patients [24, 28, 29] were examined for the prognostic role of CAR on CSS. Because of on significant heterogeneity (*I*^2^ = 0, P = 0.919) was detected, a fixed-effects model was applied (Fig 3 and Table 2). The pooled HR and 95%CI were: HR = 1.65, 95%CI = 1.21–2.25, p = 0.002, which suggested high CAR predicted worse CSS in GC. The subgroup analysis showed that the elevated pretreatment CAR persistently correlated with poor CSS in various subgroups (Table 2).

**Fig 3:** Forest plot of CAR in predicting CSS of patients with GC. (A) The whole patients group; (B) The subgroup analysis by country; (C) The subgroup analysis by treatment; (D) The subgroup analysis by cut-off value; and (E) The subgroup analysis by TNM stage.

### Relationship between CAR and clinicopathological features

To further investigate the prognostic value of CAR in clinical practice, the association between CAR and 6 clinicopathological factors were analyzed. A total of 3 studies consisting 850 patients [22, 23, 25] provided the data. As shown in Fig 4A–4F and Table 3, forest plots showed that high CAR was significantly associated with male sex (OR = 1.80, 95%CI = 1.31–2.47, p<0.001), advanced tumor stage (OR = 2.14, 95%CI = 1.48–3.09, p<0.001), and tumor size ≥3cm (OR = 2.69, 95%CI = 1.84–3.93, p<0.001). However, there was no significant correlation between CAR and age (OR = 1.44, 95%CI = 0.89–2.33, p = 0.141), tumor location (OR = 0.86, 95%CI = 0.40–1.81, p = 0.682), or platelets counts (OR = 2.40, 95%CI = 0.67–8.56, p = 0.179) (Fig 4 and Table 3).

**Fig 4:** Association between CAR levels with clinicopathological characteristics of patients with GC. (A) Sex, (B) Age, (C) Tumor location, (D) Platelets counts, (E) TNM stage, and (F) Tumor size.

**Table 3:** Association between high levels of CAR and clinicopathological characteristics of patients with GC.

Clinicopathological parameters	No. of studies	No. of patients	OR (95%CI)	p	Heterogeneity		Effects model
					*I*^2^(%)	Ph	
Sex (male vs female)	3	850	1.80(1.31–2.47)	<0.001	0	0.646	Fixed
Age (≥median vs < median)	3	850	1.44(0.89–2.33)	0.141	61.4	0.075	Random
Tumor location (proximal vs remote and other)	3	850	0.86(0.40–1.81)	0.682	82.7	0.003	Random
Platelets counts (≥median vs < median)	2	513	2.40(0.67–8.56)	0.179	75.2	0.045	Random
TNM stage (III-IV vs I-II)	2	592	2.14(1.48–3.09)	<0.001	36.3	0.210	Fixed
Tumor size (cm) (≥3 vs <3)	2	592	2.69(1.84–3.93)	<0.001	24.7	0.249	Fixed

RETRACTED

### Publication bias

Potential publication bias was evaluated by using Begg’s funnel plot. As shown in Fig 5A and 5B, the funnel plot was symmetric and no significant publication bias was detected (p = 0.133 for OS and p = 1 for CSS).

**Fig 5:** Begg’s test for publication bias examination. (A) OS: p = 0.133, and (B) CSS: p = 1.

## Discussion

As an inflammatory parameter reflecting the immune responses and nutritional condition of patients, CAR was extensively explored as a prognostic marker in GC. The results regarding the association between CAR and survival outcomes were inconsistent according to previous studies. In the present meta-analysis, we synthetized data of 8 studies with 3,216 patients and found that high CAR was significantly associated with poor OS and CSS. In addition, the prognostic value of CAR was persistent in different subgroups of country, treatment, and cut-off value. We also identified the positive correlation between CAR and male sex, advanced tumor stage, and larger tumor size. Our meta-analysis demonstrated that CAR was an effective and reliable prognostic factor and a risk factor of tumor progression for patients with GC.

Recent evidence has shown the relationship between chronic inflammation and cancer in past decades [32, 33]. CRP is an acute phase protein and the production of CRP is independently mediated by interleukin 6 (IL-6) in liver. Recent studies have revealed that CRP can produce inflammatory cytokines and chemokines to facilitate cancer progression [34]. Moreover, albumin can reflect the nutrition status of host and decreased serum albumin levels are indicators of chronic diseases and malnutrition in cancer patients [35]. Therefore, CAR is a promising inflammation-based prognostic parameter because it combines CRP and albumin and is more stable than either one individually. CAR is initially shown as an is an independent risk factor for mortality in septic patients [36]. Further studies reported the prognostic significance of CAR in various cancers including hepatocellular carcinoma (HCC) [17], renal cell carcinoma [18], anal carcinoma [37], and pancreatic cancer [38]. Those studies may suggest that CAR is a potential prognostic biomarker in solid tumors.

Previous meta-analyses have explored the prognostic value of CAR in a variety of cancer [15]. A meta-analysis based on 23 studies suggests that elevated level of serum CAR predicts worse survival and unfavorable clinical characteristics in cancer patients [15]. Another meta-analysis on esophageal cancer (EC) also indicates that high pretreatment CAR is an adverse prognostic factor for EC patients, based on data of 8 studies with 2255 patients [39]. A recent meta-analysis comprising 9 studies also demonstrates that elevated pretreatment CAR is associated with poor OS and disease-free survival (DFS)/relapse-free survival (RFS) in colorectal cancer (CRC). In addition, high CAR is also correlated with several clinical features in patients with CRC [20]. In the present meta-analysis, we showed the prognostic impact of CAR and its potential application as a risk factor in GC. Our results were in accordance with findings of previous meta-analyses of other cancer types [15, 20, 39]. In combination with other studies, we propose that CAR could be a novel and promising prognostic factor in cancer patients, especially gastrointestinal tumors including EC [39], GC, CRC [20], pancreatic cancer, and HCC [40].

RETRACTED

We noticed that a meta-analysis on the prognostic value of CAR in GC was published very recently [41]. The work conducted by Yang and colleagues was elegant and they included 8 observational studies with 3102 patients in meta-analysis and reported that a high pretreatment CAR was significantly associated with poor survival for patients with GC [41]. When our meta-analysis was prepared, Yang’s work was not published, and our study was the first meta-analysis exploring the prognostic value of CAR in GC at that time. We applauded for Yang’ s study; and those findings are important. However, our meta-analysis was different and provided additional information, compared with Yang’s work [41]. The novelty and strengths of our meta-analysis are highlighted in the following aspects. First, we provided additional and important findings. In our meta-analysis, we analyzed the correlation between CAR and clinicopathological features in GC. We identified the positive correlation between CAR and male sex, advanced tumor stage, and larger tumor size in GC. These findings suggest that a high CAR is predictive of tumor progression, which could aid in the managements of those high-risk patients. In Yang’s study [41], those analyses were not reported. Second, the included studies in our meta-analysis and in Yang’s work were different and the eligible studies in our meta-analysis were strictly selected by uniform inclusion and exclusion criteria, which guaranteed the credibility of the results. For example, we noticed that a study focusing on patients with adenocarcinoma of the esophagogastric junction (AEG) and upper gastric cancer (UGC) [42] was included in Yang’s meta-analysis. However, we excluded this study [42] after full-text examination because this study focused on patients with AEG and UGC, other than GC.

RETRACTED

The cut-off value is important to identify patients with high or low CAR, therefore, the identifying of cut-off values could influence the subgroup of patients. Notably, the cut-off values are different in included studies for OS and CSS analysis. The investigators used various methods to determine the optimal cut-off value of CAR, including operating characteristics (ROC) curve and median value. In the subgroup analysis of the meta-analysis, both CAR<0.2 and CAR≥0.2 showed significant prognostic efficiency. We suggest that a uniform optimal cut-off value of CAR should be applied for GC in future researches.

Several limitations still should be acknowledged in the present meta-analysis. First, most of the included studies (7 out of 8) are retrospective cohort studies, which may increase the risk of selection bias. Second, the sample size was relatively small. Only 6 studies and 3 studies are included for the analysis of OS and CSS, the number of included studies and subjects was limited. Third, the cut-off values to identify high CAR levels were different in included studies. These diverse thresholds could lead to inconsistent recruitment of patients and cause heterogeneity among studies. Fourth, the sample size for the correlation of CAR and clinicopathological factors were relatively small. Only 3 studies with 850 cases were included, which may lead to selection bias in this meta-analysis.

## Conclusions

In summary, elevated pretreatment CAR is a prognostic marker of poor OS and CSS in patients with GC. Furthermore, high CAR levels are associated with clinicopathological features reflecting tumor progression. Thus, CAR has the potential to be applied as a useful marker for prognostication and identification of high-risk patients with GC. Considering several limitations to this meta-analysis, more large-scale clinical trials are still needed to confirm our results.

## Supporting information

S1 Checklist PRISMA checklist. (DOC)

S1 Table The details of the NOS scale for included studies in this meta-analysis. (DOCX)

## References

[1] Van CutsemE, SagaertX, TopalB, HaustermansK, PrenenH. Gastric cancer. Lancet. 2016;388(10060):2654–64. Epub 2016/05/10. 10.1016/S0140-6736(16)30354-3 .27156933

[2] BrayF, FerlayJ, SoerjomataramI, SiegelRL, TorreLA, JemalA. Global cancer statistics 2018: GLOBOCAN estimates of incidence and mortality worldwide for 36 cancers in 185 countries. CA: a cancer journal for clinicians. 2018;68(6):394–424. Epub 2018/09/13. 10.3322/caac.21492 .30207593

[3] LyonsK, LeLC, PhamYTH, BorronC, ParkJY, TranCTD, et al. Gastric cancer: epidemiology, biology, and prevention: a mini review. European Journal of Cancer Prevention. 2019;28(5):397–412. 10.1097/CEJ.0000000000000480 PubMed PMID: WOS:000498558800003. 31386635

RETRACTED

[4] CharalampakisN, EconomopoulouP, KotsantisI, ToliaM, SchizasD, LiakakosT, et al. Medical management of gastric cancer: a 2017 update. Cancer Medicine. 2018;7(1):123–33. 10.1002/cam4.1274 PubMed PMID: WOS:000425822300013. 29239137PMC5773977

[5] LasithiotakisK, AntoniouSA, AntoniouGA, KaklamanosI, ZorasO. Gastrectomy for Stage IV Gastric Cancer. A Systematic Review and Meta-analysis. Anticancer Research. 2014;34(5):2079–85. PubMed PMID: WOS:000335545900003. 24778009

[6] KonoK, NakajimaS, MimuraK. Current status of immune checkpoint inhibitors for gastric cancer. Gastric cancer: official journal of the International Gastric Cancer Association and the Japanese Gastric Cancer Association. 2020;23(4):565–78. 10.1007/s10120-020-01090-4 PubMed PMID: WOS:000536066900001. 32468420

[7] BebnowskaD, GrywalskaE, Niedzwiedzka-RystwejP, Sosnowska-PasiarskaB, Smok-KalwatJ, PasiarskiM, et al. CAR-T Cell Therapy-An Overview of Targets in Gastric Cancer. Journal of Clinical Medicine. 2020;9(6). 10.3390/jcm9061894 PubMed PMID: WOS:000552493700001. 32560392PMC7355670

[8] ZhouC, ZhongX, SongYX, ShiJX, WuZH, GuoZX, et al. Prognostic Biomarkers for Gastric Cancer: An Umbrella Review of the Evidence. Frontiers in Oncology. 2019;9. 10.3389/fonc.2019.00009 PubMed PMID: WOS:000502743100001. 31850212PMC6895018

[9] DiakosCI, CharlesKA, McMillanDC, ClarkeSJ. Cancer-related inflammation and treatment effectiveness. Lancet Oncology. 2014;15(11):E493–E503. 10.1016/S1470-2045(14)70263-3 PubMed PMID: WOS:000343096800030. 25281468

[10] YangY, GaoP, SongY, SunJ, ChenX, ZhaoJ, et al. The prognostic nutritional index is a predictive indicator of prognosis and postoperative complications in gastric cancer: A meta-analysis. Ejso. 2016;42(8):1176–82. 10.1016/j.ejso.2016.05.029 PubMed PMID: WOS:000383005000011. 27293109

[11] LiJ, XuR, HuDM, ZhangY, GongTP, WuXL. Prognostic Nutritional Index Predicts Outcomes of Patients after Gastrectomy for Cancer: A Systematic Review and Meta-Analysis of Nonrandomized Studies. Nutr Cancer. 2019;71(4):557–68. Epub 2019/02/23. 10.1080/01635581.2019.1577986 .30793968

[12] AllinKH, NordestgaardBG. Elevated C-reactive protein in the diagnosis, prognosis, and cause of cancer. Critical Reviews in Clinical Laboratory Sciences. 2011;48(4):155–70. 10.3109/10408363.2011.599831 PubMed PMID: WOS:000296283100001. 22035340

[13] LiW, LuoX, LiuZ, ChenY, LiZ. Prognostic value of C-reactive protein levels in patients with bone neoplasms: A meta-analysis. PloS one. 2018;13(4):e0195769-e. 10.1371/journal.pone.0195769 .29668751PMC5906001

RETRACTED

[14] FangY, XuC, WuP, ZhangL-H, LiD-W, SunJ-H, et al. Prognostic role of C-reactive protein in patients with nasopharyngeal carcinoma: A meta-analysis and literature review. Medicine. 2017;96(45):e8463-e. 10.1097/MD.0000000000008463 .29137033PMC5690726

[15] WuJ, TanW, ChenL, HuangZ, MaiS. Clinicopathologic and prognostic significance of C-reactive protein/albumin ratio in patients with solid tumors: an updated systemic review and meta-analysis. Oncotarget. 2018;9(17):13934–47. Epub 2018/03/24. 10.18632/oncotarget.24172 29568406PMC5862627

[16] MiyamotoT, FujitaniM, FukuyamaH, HatanakaS, KoizumiY, KawabataA. The C-Reactive Protein/Albumin Ratio Is Useful for Predicting Short-Term Survival in Cancer and Noncancer Patients. Journal of Palliative Medicine. 2019;22(5):532–7. 10.1089/jpm.2018.0404 PubMed PMID: WOS:000467304800012. 30570426

[17] KinoshitaA, OnodaH, ImaiN, IwakuA, OishiM, TanakaK, et al. The C-Reactive Protein/Albumin Ratio, a Novel Inflammation-Based Prognostic Score, Predicts Outcomes in Patients with Hepatocellular Carcinoma. Annals of Surgical Oncology. 2015;22(3):803–10. 10.1245/s10434-014-4048-0 PubMed PMID: WOS:000350553100018. 25190127

[18] TsujinoT, KomuraK, HashimotoT, MuraokaR, SatakeN, MatsunagaT, et al. C-reactive protein-albumin ratio as a prognostic factor in renal cell carcinoma—A data from multi-institutional study in Japan. Urologic Oncology-Seminars and Original Investigations. 2019;37(11). 10.1016/j.urolonc.2019.04.002 PubMed PMID: WOS:000492676200010. 31053528

[19] WangY, HuX, HuangY, XuWY, WuYM, LiPF, et al. Prognostic value of the C-reactive protein to albumin ratio in esophageal cancer: A systematic review and meta-analysis. The Kaohsiung journal of medical sciences. 2019. Epub 2019/09/13. 10.1002/kjm2.12129 .31512813PMC11896523

[20] ZhouQP, LiXJ. C-Reactive Protein to Albumin Ratio in Colorectal Cancer: A Meta-Analysis of Prognostic Value. Dose-response: a publication of International Hormesis Society. 2019;17(4):1559325819889814. Epub 2019/12/05. 10.1177/1559325819889814 31798355PMC6868585

[21] SunF, GeX, LiuZ, DuS, AiS, GuanW. Postoperative C-reactive protein/albumin ratio as a novel predictor for short-term complications following gastrectomy of gastric cancer. World J Surg Oncol. 2017;15(1):191. Epub 2017/10/27. 10.1186/s12957-017-1258-5 29065877PMC5655858

[22] LiuXC, SunXW, LiuJJ, KongPF, ChenSX, ZhanYQ, et al. Preoperative C-Reactive Protein/Albumin Ratio Predicts Prognosis of Patients after Curative Resection for Gastric Cancer. Translational Oncology. 2015;8(4):339–45. 10.1016/j.tranon.2015.06.006 PubMed PMID: WOS:000360276400013. 26310380PMC4562973

RETRACTED

[23] NiXF, WuJ, JiM, ShaoYJ, ZhouWJ, JiangJT, et al. Prognostic value of C-reactive protein/albumin ratio in patients receiving first-line palliative chemotherapy with unresectable stage IV gastric cancer. International Journal of Clinical and Experimental Pathology. 2016;9(12):12785–96. PubMed PMID: WOS:000390406200067.

[24] ToiyamaY, ShimuraT, YasudaH, FujikawaH, OkitaY, KobayashiM, et al. Clinical Burden of C-Reactive Protein/Albumin Ratio Before Curative Surgery for Patients with Gastric Cancer. Anticancer Res. 2016;36(12):6491–8. Epub 2016/12/07. 10.21873/anticanres.11248 .27919972

[25] MaoM, WeiX, ShengH, ChiP, LiuY, HuangX, et al. C-reactive protein/albumin and neutrophil/lymphocyte ratios and their combination predict overall survival in patients with gastric cancer. Oncol Lett. 2017;14(6):7417–24. Epub 2018/01/19. 10.3892/ol.2017.7179 29344182PMC5755031

[26] SaitoH, KonoY, MurakamiY, ShishidoY, KurodaH, MatsunagaT, et al. Prognostic Significance of the Preoperative Ratio of C-Reactive Protein to Albumin and Neutrophil-Lymphocyte Ratio in Gastric Cancer Patients. World journal of surgery. 2018;42(6):1819–25. Epub 2017/12/23. 10.1007/s00268-017-4400-1 .29270656

[27] ToyokawaT, MugurumaK, TamuraT, SakuraiK, AmanoR, KuboN, et al. Comparison of the prognostic impact and combination of preoperative inflammation-based and/or nutritional markers in patients with stage II gastric cancer. Oncotarget. 2018;9(50):29351–64. Epub 2018/07/24. 10.18632/oncotarget.25486 30034622PMC6047670

[28] LiuXC, WuZM, LinEZ, LiW, ChenYB, SunXW, et al. Systemic prognostic score and nomogram based on inflammatory, nutritional and tumor markers predict cancer-specific survival in stage II-III gastric cancer patients with adjuvant chemotherapy. Clinical Nutrition. 2019;38(4):1853–60. 10.1016/j.clnu.2018.07.015 PubMed PMID: WOS:000473381200046. 30075998

[29] LuJ, XuBB, ZhengZF, XieJW, WangJB, LinJX, et al. CRP/prealbumin, a novel inflammatory index for predicting recurrence after radical resection in gastric cancer patients: post hoc analysis of a randomized phase III trial. Gastric cancer: official journal of the International Gastric Cancer Association and the Japanese Gastric Cancer Association. 2019;22(3):536–45. Epub 2018/11/01. 10.1007/s10120-018-0892-0 .30377862

[30] MoherD, LiberatiA, TetzlaffJ, AltmanDG, GrpP. Preferred Reporting Items for Systematic Reviews and Meta-Analyses: The PRISMA Statement. Journal of Clinical Epidemiology. 2009;62(10):1006–12. 10.1016/j.jclinepi.2009.06.005 PubMed PMID: WOS:000270250500003. 19631508

[31] StangA. Critical evaluation of the Newcastle-Ottawa scale for the assessment of the quality of nonrandomized studies in meta-analyses. European Journal of Epidemiology. 2010;25(9):603–5. 10.1007/s10654-010-9491-z PubMed PMID: WOS:000282102200001. 20652370

RETRACTED

[32] ChenDS, MellmanI. Elements of cancer immunity and the cancer-immune set point. Nature. 2017;541(7637):321–30. 10.1038/nature21349 PubMed PMID: WOS:000396128800030. 28102259

[33] GrivennikovSI, GretenFR, KarinM. Immunity, Inflammation, and Cancer. Cell. 2010;140(6):883–99. 10.1016/j.cell.2010.01.025 PubMed PMID: WOS:000275746600012. 20303878PMC2866629

[34] AsegaonkarSB, AsegaonkarBN, TakalkarUV, AdvaniS, ThoratAP. C-Reactive Protein and Breast Cancer: New Insights from Old Molecule. International Journal of Breast Cancer. 2015. 10.1155/2015/145647 PubMed PMID: WOS:000215219100004. 26693355PMC4674617

[35] Onate-OcanaLF, Aiello-CrocifoglioV, Gallardo-RinconD, Herrera-GoepfertR, Brom-ValladaresR, CarrilloJF, et al. Serum albumin as a significant prognostic factor for patients with gastric carcinoma. Annals of Surgical Oncology. 2007;14(2):381–9. 10.1245/s10434-006-9093-x PubMed PMID: WOS:000243765500016. 17160496

[36] RanzaniOT, ZampieriFG, ForteDN, AzevedoLCP, ParkM. C-Reactive Protein/Albumin Ratio Predicts 90-Day Mortality of Septic Patients. Plos One. 2013;8(3). 10.1371/journal.pone.0059321 PubMed PMID: WOS:000316252500080. 23555017PMC3595283

[37] MartinD, RodelF, BalermpasP, WinkelmannR, FokasE, RodelC. C-Reactive Protein-to-Albumin Ratio as Prognostic Marker for Anal Squamous Cell Carcinoma Treated With Chemoradiotherapy. Frontiers in Oncology. 2019;9. 10.3389/fonc.2019.00009 PubMed PMID: WOS:000498911800001. 31788452PMC6856140

[38] LiuZQ, JinKZ, GuoM, LongJ, LiuL, LiuC, et al. Prognostic Value of the CRP/Alb Ratio, a Novel Inflammation-Based Score in Pancreatic Cancer. Annals of Surgical Oncology. 2017;24(2):561–8. 10.1245/s10434-016-5579-3 PubMed PMID: WOS:000391926600037. 27650825

[39] LiuZ, ShiH, ChenL. Prognostic role of pre-treatment C-reactive protein/albumin ratio in esophageal cancer: a meta-analysis. BMC Cancer. 2019;19(1):1161. Epub 2019/12/01. 10.1186/s12885-019-6373-y .31783812PMC6884775

[40] FanY, GuX, GaoZ. Prognostic value of C-reactive protein to albumin ratio in patients with hepatocellular carcinoma: A meta-analysis. Clin Res Hepatol Gastroenterol. 2019. Epub 2019/08/25. 10.1016/j.clinre.2019.07.014 .31444039

[41] YangX, SongX, ZhangL, WuC. Prognostic role of the pretreatment C-reactive protein/albumin ratio in gastric cancer: A systematic review and meta-analysis. Medicine (Baltimore). 2020;99(10):e19362. Epub 2020/03/10. 10.1097/MD.0000000000019362 .32150079PMC7478778

[42] KudouK, SaekiH, NakashimaY, KamoriT, KawazoeT, HarutaY, et al. C-reactive protein/albumin ratio is a poor prognostic factor of esophagogastric junction and upper gastric cancer. Journal of Gastroenterology and Hepatology. 2019;34(2):355–63. 10.1111/jgh.14442 PubMed PMID: WOS:000459628400011. 30119141

